The article "Koebner phenomenon leading to the formation of new psoriatic lesions: evidences and mechanisms" was published in 2019. Journal: Biosci Rep.

# Koebner phenomenon leading to the formation of new psoriatic lesions: evidences and mechanisms

**DOI:** 10.1042/BSR20193266

**Published:** 2019-12-04

**Authors:** Yong-Zhi Ji, Shi-Rui Liu

**Affiliations:** Department of Dermatology, Second Hospital of Jilin University, Changchun, China

**Keywords:** cytokines, immune system, Koebner phenomenon, psoriasis, tryptase

## Abstract

Koebner phenomenon refers to the emergence of new psoriatic lesions in the healthy skin regions following an injury/trauma to psoriatic patients. The occurrence of psoriatic lesions at unusual areas of the body regions such as on penis, around eyes and on keloids suggest that the Koebner phenomenon may be responsible for these lesions. A number of agents/triggers have been reported to induce the development of new psoriatic lesions in healthy skin areas and these include, tattooing skin, radiations, skin incision, viral infections and striae etc. The different mechanisms that contribute in inducing the development of new psoriatic lesions as Koebernization include the involvement of mast cell-derived inflammatory mediators such as tryptase, IL-6, IL-8, IL-17, and IL-36γ. Moreover, an increased expression of nerve growth factor (NGF) and vascular endothelial growth factor (VEGF) also contribute in Koebernization. Apart from these, there is a critical role of α 2 β1 integrins, S100A7 (psoriasin) and S100A15 (koebnerisin), change in the ratio of CD4^+^/CD8^+^ T cells, down-regulation of mechanosensitive polycystin 1 protein, decrease in inflammation controlling atypical chemokine receptor 2 (ACKR2), reduced expression of N-methyl-d-aspartate (NMDA) receptors (NMDARs) on the keratinocytes and increase in levels of chemokines (CXCL8 and CCL20) in inducing formation of new psoriatic lesions. The present review discusses the role of Koebner phenomenon in the development of new psoriatic lesions. Moreover, it also describes the mechanisms involved in Koebernization in the form of discussion of different key targets that may be potentially modulated pharmacologically to attenuate/halt the development of new psoriatic lesions.

## Introduction

Heinrich Koebner (1838–1904) reported the emergence of new psoriatic lesions in the non-involved (healthy) skin region following an injury/trauma to the healthy skin areas of psoriatic patients [1]. Thereafter, many scientists identified the occurrence of new psoriatic lesions in approximately 25–30% of patients in the uninvolved skin region following the injury in that skin region [2,3]. Under experimental conditions also, mild skin injury (pricking, tape stripping or punch biopsy) has been shown to induce psoriatic plaques (erythematous papules) in approximately 25% of psoriatic patients [4,5]. The Koebner phenomenon has also been described in other skin diseases including vitiligo, lichen planus, viral warts, and molluscum contagiosum etc [6–8]. Different triggers including drugs, chronic pressure on the skin, solar exposure, cutaneous trauma, and hot water burn are reported to induce the development of papulopustular eruptions through activation of Koebner phenomenon [9,10].

Nevertheless, the Koebner phenomenon is best described in association with psoriasis and there have been a number of studies showing the association of Koebnerization with psoriasis [11,12]. The occurrence of psoriatic lesions at unusual areas of the body regions such as on penis, around eyes, and on keloids suggest that the Koebner phenomenon may be responsible for these psoriatic lesions [13–15]. Moreover, the development of dactylitis (inflammation of an entire digit, finger, or toe) in psoriatic arthritis has been linked with deep Koebner phenomenon of the flexor tendon-associated accessory pulleys [16]. Indeed, a number of agents/triggers have been reported to induce the development of new psoriatic lesions in healthy skin areas and these include, tattooing skin, radiations, skin incision, viral infections, and striae etc [17–19]. The different mechanisms that may possibly contribute in inducing the development of new psoriatic lesions as Koebernization include the involvement of mast cell-derived inflammatory mediators [20–22], nerve growth factor (NGF) and its receptor system [23], vascular endothelial growth factor (VEGF) [24], α 2 β1 integrins [25], S100A7 (psoriasin) and S100A15 (koebnerisin) [26], increase in the ratio of CD4^+^/CD8^+^ T cells [5], down-regulation of polycystins [27], down-regulation of atypical chemokine receptor 2 (ACKR2) [28], decreased expression of N-methyl-d-aspartate (NMDA) receptor (NMDAR) on the keratinocytes [29] and increase in chemokines [30]. The present review discusses the role of Koebner phenomenon in the development of new psoriatic lesions at the healthy body parts in response to an injury with possible mechanisms.

## The occurrence of psoriatic lesion at uncommon body parts suggests the role of Koebner phenomenon

The occurrence of psoriatic lesions in the body parts, which are not usually affected by psoriasis suggests that Koebner reaction may be responsible for the development of psoriatic lesions at the unusual body regions. A patient showing the development of a rare type of psoriasis on the penis following oral-genital exposure is an indication of Koebner reaction [31]. The development of pustular psoriasis over the keloids and new psoriatic lesions on the site of healing/healed herpes zoster lesions (shingles) also suggest that Koebner phenomenon may be responsible for these psoriatic lesions [13,14,32–34]. The development of periocular psoriasis in the form of blepharitis and conjunctivitis following an external dacryocystorhinostomy [15] and psoriasis at gastrostomy tube site [35] suggest the role of Koebner reaction in the development of psoriatic lesions. Vitiligo and psoriasis are two different skin diseases with different etiology and pathogenesis. However, in some patients, psoriatic plaques are confined to the vitiliginous areas of the skin, with no involvement of the normal skin. This sort of anatomical coexistence of psoriasis and vitiligo may be possibly due to the Koebner phenomenon [36,37].

## Agents that may trigger new psoriatic lesions in uninvolved skin area as a Koebner reaction

The Koebner phenomenon in psoriasis is a common response to skin trauma/injury, may be mild or severe [38] and there is a long list of agents that may trigger the development of new psoriatic lesion as a part of Koebner phenomenon. There has been an exponential increase in the decorative tattooing as body art in the last two decades. However, a large number of studies have shown the development of new psoriatic lesions after tattooing skin as a Koebner reaction [18,39–43]. The other factors/agents that are reported to exacerbate psoriasis as Koebner reaction include megavoltage irradiations [44], radiotherapy for carcinoma of breast [45], exposure to purified protein derivative (PPD)/Mantoux test [46,47], surgical incision during breast reconstruction [19,48], needle acupuncture [49], prosthesis after amputation of the leg [50], secondary syphilis [51], cupping therapy, a traditional Chinese medicine [52,53], striae distensae and striae gravidarum [17,54], ECG [55], itching (one of the core features of psoriasis)-induced skin injury [56], and viral infection-induced hand-foot-and-mouth disease [57].

## Disruption/injury to the epidermis is critical, but not sufficient alone to induce new psoriatic lesions

It has been shown that the disruption of a functional and structural permeability barrier is critical for the appearance of psoriasis as Koebner reaction [58]. Accordingly, the importance of the rupturing of the epidermis in initiating the Koebner response has been well documented [59]. Along with it, an important role of secondary dermal reactions in the development of psoriatic lesions at the site of injury has also been defined. In a clinical experimental study, it was shown that the incidences of development of new psoriatic lesions were much higher, when the skin injury was induced using low-pressure suction (to induce suction blisters) and the top of blisters was removed and left unoccluded (9 as Koebner-positive out of 14 patients). In contrast, the incidences of Koebner reaction were very low in cellotape stripping-induced superficial injury (8 as Koebner-positive out of 37 patients), which only induces superficial injury to epidermis without significant involvement of underlying dermis [60]. It suggests that the superficial damage to the epidermis may be an initiating event; however, subsequent reactions in the dermal region are also important in the development of new lesions as Koebner reaction.

## Keratinocytes are more committed to terminally differentiate in Koebner-positive patients

The presence of Ulex europaeus agglutinin (UEA I) binding sites on the cells is commonly employed as a marker for terminal differentiation [61]. Using the UEA I binding site as a biomarker of terminal differentiation, the study of Heng et al. [62] demonstrated that the keratinocytes present in the stratum spinosum are more committed to terminally differentiate in Koebner-positive patients and those patients, who are more prone to develop secondary psoriatic lesions following tape-stripping. Indeed, the authors demonstrated the increased number of UEA I binding sites of l-Fucose in the stratum spinosum of the epidermis portion (detected after biopsy studies) in the healthy (uninvolved) skin area in the psoriatic patients, who were more prone to develop Koebner reaction. The authors also correlated the expression of UEA I binding sites and l-Fucose moiety on the keratinocytes of stratum spinosum in 7-day post-tape-stripping and 8-week biopsies to a moderate and marked increase in the proliferative index, respectively. In contrast, the UEA I binding sites were not expressed on keratinocytes in the biopsies of Koebner-negative and non-psoriatic individuals [62]. It suggests that the functional changes in the keratinocytes (in terms of their commitment to terminal differentiation) may be an important factor in inducing Koebner-positive or Koebner-negative state in psoriatic patients.

## Possible mechanisms contributing to Koebernization in psoriatic patients

Scientists have attempted to explore the different mechanisms that may contribute to induce the development of new psoriatic lesions as Koebernization:

### Mast cells

Skin resident mast cells have a detrimental effect on different inflammatory skin diseases including psoriasis [63,64] and hence, selective reduction in the number or activity of mast cells has been proposed to overcome the symptoms of psoriasis. Mast cells release a myriad of primary and secondary inflammatory mediators [65]. However, the mediators with a significant role in the Koebner phenomenon are discussed below (Figure 1):

**Figure 1:** Representation of the role of mast cells-derived mediators in inducing the formation of new psoriatic lesions Tryptase may directly act as a mitogen to increase the proliferation of epithelial cells and dermal fibroblasts. Moreover, tryptase may activate PAR-2 receptors located on the mast cells to induce its activation, thus leading to the initiation of the self-amplification process. In response, the activated mast cells release IL-8, which contributes to the inflammatory process. The psoriatic keratinocytes act in concert with the mast cells to potentiate the inflammation in different ways including the release of IL-33 from the keratinocytes, which activate the mast cells to release IL-6. Furthermore, TLR-3 released from the keratinocytes interacts with IL-17 released from the mast cells to induce the release of IL-36γ and other inflammatory mediators. Mast cell-derived IL-17 activates downstream signaling cascade involving the activation of p38MAPK and NF-kB to induce the formation of new psoriatic lesions. Abbreviations: MAPK, mitogen-activated protein kinase; PAR, proteinase-activated receptor.

#### Tryptase

There have been a large number of studies documenting the key role of tryptase in the pathogenesis of psoriasis [66–68]. Tryptase is a trypsin-like serine protease, which is released by the mast cells during skin inflammatory reactions [69]. Accordingly, it has been hypothesized that there may be an increase in the levels of tryptase following skin injury/trauma [70], which may contribute to the development of psoriatic lesions as Koebner reaction [20]. The precise mechanisms that may lead to the development of psoriatic lesion following increase in tryptase levels are not defined. However, it is postulated that tryptase may contribute in psoriasis development by directly acting as mitogen for the epithelial cells and dermal fibroblasts [71,72]; activating proteinase-activated receptors (PAR)-2 on the mast cells to release IL-8 [73] and inducing the mast cell accumulation via a PAR-2 dependent mechanism leading to self-amplification mechanism [74].

#### IL-17, NF-kB, and signal transducer and activator of transcription 3

It has been demonstrated that the mast cells along with neutrophils, but not T cells, are the predominant cells that contain IL-17 in the human skin [75] and IL-17 is one of the principal cytokines involved in the pathogenesis of psoriasis [76,77]. Accordingly, secukinumab (anti-IL-17 monoclonal antibody) has been approved as a first-line treatment for the management of moderate-to-severe plaque psoriasis [78] and as a second-line treatment for psoriatic arthritis. Moreover, other monoclonal antibodies targeting IL-17 including ixekizumab and brodalumab have also been approved by the FDA for the treatment of plaque psoriasis [79,80]. Apart from the role of IL-17 in psoriasis, its role has also been described in injury-induced keratinocyte activation, an important pathogenic step in Koebner phenomenon. It has been shown that IL-17A synergizes with TLR3 (released from the necrotic keratinocytes) in activating keratinocytes and increasing the release of IL-36γ and other proinflammatory mediators. IL-17A and TLR3-mediated synergistic up-regulation of IL-36γ and other pro-inflammatory mediators were inhibited in the presence of siRNA of IκBζ and blockers of p38 mitogen-activated protein kinase (MAPK) and NF-κB. It suggests that IL-17A-mediated inflammatory actions in Koebner phenomenon are dependent on the activation of p38 MAPK and NF-κB [21]. Indeed, NF-kB has been reported as a key transcriptional factor of psoriasis [81,82] and different pharmacological agents including quercetin and BAY 11-7082 are shown to inhibit the development of psoriatic lesion by inhibiting the activation of this transcriptional factor [83].

Signal transducer and activator of transcription 3 (STAT3) is a transcriptional factor, which is linked with survival, proliferation, and angiogenesis [84]. There has been a very recent study describing the key role of STAT3 in regulating the functionality of IL-17 producing γδ T (γδT17) cells. Indeed, it was shown that there is a decrease in the expression of IL-17 in mice lacking STAT3 expression in γδT17 cells. Moreover, these mice also failed to develop psoriasis-like inflammation suggesting the essential role of STAT3 in the production of inflammatory cytokines and development of psoriatic lesions [85]. The key role of STAT3 in the development of psoriatic lesion is further supported by a study showing that treatment with ustekinumab (a monoclonal antibody that targets IL-12 and IL-23 and is used clinically for psoriasis) down-regulates the expression of STAT3 in psoriatic patients [86].

#### IL-6

IL-6 is another important cytokine released by the mast cells [87] and the role of IL-6 has also been well documented in the pathogenesis of psoriasis [88]. Moreover, a research study has shown an increase in IL-6 immunoreactivity in biopsies from Köebner-positive patients in comparison with Köebner-negative patients. Indeed, the Köebner reaction was induced in uninvolved psoriatic skin using the tape-stripping method and biopsies were collected up to 7 days for histochemical analysis. Along with the rise in IL-6 immunoreactivity, an increase in the number of IL-33^+^ cells was also reported in Köebner-positive dermal skin at days 3–7 suggesting the key role of IL-6 and IL-33 in Koebner reaction [22]. IL-33 is an important cytokine, whose release has been reported from the psoriatic keratinocytes and IL-33 stimulates the mast cells to release proinflammatory mediators including IL-6 [89].

### NGF and its receptor system

NGF is a neurotrophic molecule and at the skin level, it is synthesized by the keratinocytes, mainly in response to histamine release [90]. Although its normal function is to stimulate the sprouting of nerve fibers, yet its key role in inducing neurogenic inflammation in several inflammatory dermatoses, including psoriasis has also been described [91,92]. It is suggested that NGF released from keratinocytes acts on the NGF receptors, p75 neurotrophin receptor (p75NTR) and tyrosine kinase A (TrkA) present on the keratinocytes to induce keratinocyte proliferation in an autocrine manner [93]. Moreover, NGF contributes to induce neuroinflammation by up-regulating the levels of neuropeptides (substance P and calcitonin gene-related protein) and increasing chemokine expression on the keratinocytes [94]. The key role of NGF-p75NTR-TrkA was further substantiated by the reports showing the efficacy of K252a, a high-affinity NGF receptor blocker, in improving psoriasis in transplanted psoriatic plaques in the SCID mice [95]. Moreover, the study of Raychaudhuri et al. [23] demonstrated the key role of NGF in the development of Koebner-induced psoriatic plaques. The authors reported the marked up-regulation of NGF in Koebner-positive lesions 24 h after skin trauma by the tape-stripping method, which reached its maximum level in the second week. Moreover, the cultured keratinocytes isolated from the non-lesional skin of psoriatic patients produced higher levels of NGF (approximately ten-times) in comparison with keratinocytes isolated from healthy individuals. These findings were further supported by the results showing that transplantation of psoriatic plaque in SCID-human skin xenograft model led to marked proliferation of NGF receptor-positive nerve fibers as compared with few nerves in the transplanted normal human skin [23].

### VEGF

Research studies have documented that psoriasis is an angiogenesis-dependent disease and a high expression of angiogenesis promoting factor, i.e. VEGF in the skin portion is linked with the pathogenesis of psoriasis. Accordingly, inhibitors of VEGF have been exploited as potential agents in controlling the development of psoriasis [96,97]. Moreover, it has also been shown that the excessive protein expression of epidermal VEGF-A is important in promoting angiogenesis and epidermal hyperplasia observed during Koebner (isomorphic) phenomenon in response to injury in psoriatic patients. In repeated tape stripping, a model of psoriasiform hyperplasia, the mRNA and protein expression of VEGF-A was up-regulated in the normal hairless mice. However, epidermal VEGF^(−/−)^ mice exhibited a decrease in VEGF signaling, a decrease in the number of dermal capillaries with reduced vascular permeability, reduced angiogenesis and decrease in epidermal hyperplasia in response to repeated tape stripping. It suggests that in response to external trauma, excessive production of VEGF may contribute to the development of excessive angiogenesis and epidermal hyperplasia, which may be an important contributing mechanism in the Koebner reaction during psoriasis [24].

### α 2 β1 integrin

Within the skin, the expression of α 2 β1 integrins is usually confined to the basal layer of the epidermis. However, the expression of integrins in the suprabasal layer has been linked to the hyperproliferative epidermis and psoriasis [98]. Indeed, transgenic mice with expression of α 2 β1 integrin in the suprabasal epidermal layers are shown to develop the typical features of psoriasis including epidermal hyperproliferation, perturbed keratinocyte differentiation, and skin inflammation [99]. The role of integrins in the Koebner phenomenon was described using transgenic mice expressing α 2 β1 integrin in the suprabasal epidermal layers. In normal mice, a mild epidermal wound was followed by normal healing within 14 days. However, similar type of mild epidermal wound in transgenic mice led to the development of chronic inflammation, which was very similar to the Koebner phenomenon in psoriatic patients [25]. Furthermore, it has been reported that integrins may lead to the activation of MAPKs either directly or indirectly through IL-1 to induce the development of typical features of psoriasis [100]. However, the role of integrin in activating MAPK signaling in Koebner reaction-induced psoriatic lesions needs to be explored.

### S100A7 (Psoriasin) and S100A15 (Koebnerisin)

S100 proteins are the low molecular weight proteins (9–13 kDa), which are characterized by the presence of two calcium-binding motifs. These are abundantly expressed in the epidermis including on the keratinocytes and their normal functions include regulating the cell growth, cell differentiation, and the inflammatory response [101]. S100A7 (psoriasin) and S100A15 (koebnerisin) are S100 calcium-binding proteins, which were first identified in the inflamed psoriatic skin. These two proteins are homologous, but distinct in regulation and function [102]. It has been found that inflammation-prone psoriatic skin constitutively expresses high levels of S100A7 and S100A15 in the epidermis. Moreover, it is also reported that leukocyte-derived S100A15 and S100A7 may also act as systemic mediators of inflammation in psoriasis [103]. The role of these proteins in the Koebner reaction was demonstrated in genetically modified mice with overexpression of doxycycline-regulated mS100a7a15 (mice S100A7 and S100A15) in the skin keratinocytes. Such mice exhibited an exaggerated inflammatory and immune response in response to mild exogenous injury (abrasion) in the form of Koebner reaction. The site of injury was infiltered with immune cells and exhibited the elevated concentrations of proinflammatory cytokines, which are linked to the pathogenesis of psoriasis. Mechanistically, it was reported that mS100a7a15 directly acts as a chemoattractant to increase the infiltration of leukocytes in the skin. Moreover, it was deduced that the binding of mS100a7a15 to the receptor of advanced glycation end products (RAGE) was essential for activating the immune and inflammatory response as a part of Koebner reaction [26]. The previous study of the same group of scientists also delineated that the chemotactic activity of S100A7 is mediated by its binding to RAGE and inflammatory actions were potentiated in the presence of S100A15 [104] suggesting the S100A7A15–RAGE axis as a potential therapeutic target to combat Koebner phenomenon.

### Changes in the ratio of CD4^+^/CD8^+^ cells

The changes in the immunological status are critical in the induction of inflammatory diseases such as psoriasis and an increase in the ratio of CD4^+^/CD8^+^ T cells has been found in early as well as in late phases of psoriasis [105]. In Koebner-positive patients also, a change in the ratio of CD4^+^/CD8^+^ cells has been identified in the epidermis as well as in dermis portions in untraumatized and uninvolved skin portions of psoriatic patients. Indeed, a small increase in number of CD4^+^ cells, a larger decrease in CD8^+^ cells and no significant changes in the epidermal dendritic cells have been reported in the Koebner-positive patients. It suggests that the predominance of CD4^+^ cells over the CD8^+^ T cells in the epidermis increases the tendency of uninvolved skin of the psoriatic patients to become lesional following skin trauma [5].

### Down-regulation of polycystins

Polycystins are the mechanosensitive molecules, which act as key regulators of the cellular mechanosensitivity and mechanotransduction [106,107]. Since psoriatic plaques are often found in the areas subjected to mechanical injury or trauma due to Koebner phenomenon, therefore it has been proposed that there may be a key role of mechanosensitive channels and polycystin proteins in the pathogenesis of psoriasis [108,109]. Indeed, it is reported that there is a down-regulation of polycystin 1 protein, which may be linked to the development of psoriatic lesions. In *in vitro* cellular model of psoriasis, knockout of polycystin 1 gene in HaCaT cells was associated with elevation of psoriasis-related biomarkers including cytokines. Moreover, the functional inhibition of polycystin 1 led to increased cellular proliferation and migration of HaCaT cells. In addition, it was also shown that the down-regulation of polycystin 1 in HaCaT cells leads to the activation of ERK and mTOR. More precisely, it was reported that the loss of polycystin 1 protein leads to the activation of ERK-dependent-mTOR signaling pathway activation. These *in vitro* findings were also verified in the human samples of psoriatic plaques showing the down-regulation of polycystin1, and elevation of ERK along with mTOR substrates suggesting that polycystin 1/ERK/mTOR signaling may be therapeutically exploited to reduce the occurrence of psoriatic lesions, particularly in the regions subjected to mechanical injury [27].

### Down-regulation of ACKR2

ACKR2, also named as D6, plays a vital role in controlling inflammatory reactions as these receptors serve as scavengers for proinflammatory cytokines and chemokines [110]. Due to their inflammatory regulatory functions, ACKR2 limits the spreading of psoriasiform skin inflammation to the remote body area [111]. In other words, ACKR2 functions to overcome the inflammatory process-linked with psoriasis [112]. Regarding the Koebner phenomenon, it is reported that the expression of ACKR2 is down-regulated in response to cell trauma. Along with it, tensile cell stress has been shown to rapidly down-regulate the expression of ACKR2 and concurrently, up-regulate the expression of microRNA, miR-146b. Using *in silico* and *in vitro* studies, it was shown that miR-146b directly binds to the 3′-UTR region of *ACKR2* gene, leading to decreased expression of ACKR2 in keratinocytes. Accordingly, it may be suggested that the changes in the epigenetic regulation (via miR-146b) of an atypical chemokine receptor with the down-regulation of the expression of latter protein may be responsible for the inappropriate and excessive immune response during the Koebner phenomenon in psoriasis [28].

### Down-regulation of NMDAR

Studies have shown the presence of ionotropic glutamate receptors of the NMDA type on the keratinocytes, especially in the stratum granulosum [113]. However, a significant reduction in their density in the upper epidermis has been reported in skin diseases including psoriasis. Moreover, a decrease in the expression of NMDARs has been correlated with an increase in abnormal wound healing in psoriatic patients [114]. An increase in the skin wound healing process and Koebner reaction in the psoriatic patients suggest that the proliferation of keratinocytes is not inhibited appropriately. Accordingly, scientists have explored the expression pattern of NMDARs on the keratinocytes in the presence of TNF-α, a cytokine with a prominent role in psoriasis [115]. Using gene expression analysis, the greatest reduction in the expression of NMDA-R2C was found in TNF-α-exposed keratinocytes and the apparently increased proliferation of keratinocytes was attributed to the decrease in the expression of NMDA-R2C. Accordingly, it is suggested that the non-ability of psoriatic keratinocytes to increase the expression of NMDA-R2C in response to TNF-α may contribute to increasing the proliferation of keratinocytes observed in the process of Koebernization [114].

### Chemokines

Chemokines are small molecules, which contribute to local and systemic inflammation in psoriatic patients by inducing the recruitment of T cells into psoriatic skin lesions [116]. To explore the role of chemokines in Koebner phenomenon, a very recent study has identified the changes in the cytokine/chemokine profile in *in vitro* scratched keratinocyte model. It was shown that the scratch injury on the confluent keratinocyte sheet significantly and selectively up-regulated the mRNA expression of CXCL8, CCL20, IL36G, and TNF-α. In contrast, the significant protein secretions were observed only for CXCL8 and CCL20. Moreover, the application of dexamethasone inhibited the secretion of CXCL8 and CCL20  suggesting that these chemokines may play a key role in triggering the Koebner phenomenon after scratch injury to keratinocytes [30].

## Summarized discussion

Koebner phenomenon refers to the appearance of new psoriatic lesions in non-psoriatic skin regions following an injury to that healthy area of skin [1,2,3]. The presence of psoriatic lesions in those body areas, which are not usually affected by psoriasis suggest the key role of Koebner phenomenon in spreading psoriasis [13,14,31]. There is wide variety of triggers/agents that may induce Koebernization such as irradiations [44], Mantoux test [46,47], surgical incision [19,48], needle puncture [49], prosthesis [50], secondary syphilis [51], cupping therapy [52,53], ECG [55], itching [56], and viral infections [57]. Regarding role of injury in initiating Koebernization, the deep tissue injury is more critical and superficial injury alone is not sufficient to induce the development of new psoriatic lesions [58–60]. Another interesting finding is that keratinocytes present in the stratum spinosum are more committed to terminally differentiate in Koebner-positive patients and this change in the property of keratinocytes makes the patients more susceptible to develop secondary psoriatic lesions [62]. It is essential that any sort of persistent inflammations/injurious triggers are effectively controlled; otherwise, there is a tendency to transform and develop into cancers [117–119]. Understanding the key mechanisms may help in combating the inflammatory processes including psoriatic lesions.

There has been a key role of mast cells and its mediators in inducing the formation of new psoriatic lesions. Mast cell derived-tryptase acts as a mitogen to promote the proliferation of epithelial cells and dermal fibroblasts [20,71,72], which is a critical feature in the induction of new lesion. Moreover, tryptase may activate the PAR-2 receptors located on the mast cells to activate the mast cells in an autocrine manner [73,74]. Activated mast cells may further release IL-8, which contributes to the inflammatory process [73]. There is also an important role of psoriatic keratinocytes, which act in association with the mast cells to potentiate the inflammation. Keratinocytes may release IL-33, which activate the mast cells to release IL-6 [89]. Furthermore, TLR-3 released from the keratinocytes interacts with mast cell-derived IL-17 to induce the release of IL-36γ and other inflammatory mediators [21]. Mast cell-derived IL-17 activates p38MAPK and NF-kB STAT3 signaling pathway to induce Koebernization [21]. Considering these mechanisms, it may be proposed that the pharmacological modulation of mast cells, tryptase, IL6, IL-8, IL-17, IL-33, IL-36γ, p38MAPK, and NF-kB may serve to inhibit the induction and/or progression of new psoriatic lesions following skin injury.

Scientists have also explored the role of keratinocyte-derived NGF, which acts through p75NTR and TrkA to induce keratinocyte proliferation and neuroinflammation [93–95]. Excessive formation of VEGF may lead to increased vascularization, which may also promote Koebernization [24]. Along with it, the presence of α 2 β1 integrin in the suprabasal epidermal layers (normally it is in basal epidermal layer) [98,99]; increased expression of S100A7 (psoriasin) and S100A15 (koebnerisin) in the epidermis [26]; predominance of CD4^+^ cells over the CD8^+^ T cells in the epidermis [5]; increase in chemokines viz. CXCL8 and CCL20 [30], down-regulation of mechanosensitive polycystin 1 protein [27], ACKR2 [28], and ionotropic NMDARs on the keratinocytes [114] also contribute in the development of secondary psoriatic lesions following skin injury.

## Conclusion

Koebner phenomenon is critical in inducing new (secondary) psoriatic lesions in the healthy body regions following an injury/trauma with the involvement of multiple signaling pathways including mast cell-derived tryptase, IL-6, IL-8, IL-17, IL-36γ, and other inflammatory mediators. Moreover, there is a key role of keratinocyte-derived IL-33, TLR-3, and NGF in promoting Koebernization. Excessive formation of VEGF, presence of α 2 β1 integrin in the suprabasal epidermal layers, increased expression of psoriasin and koebnerisin in the epidermis, predominance of CD4^+^ cells over the CD8^+^ T cells, increase in CXCL8 and CCL20 (chemokines), down-regulation of polycystin 1, ACKR2 and ionotropic NMDARs are other mechanisms that contribute to Koebernization. Accordingly, these targets may be pharmacologically modulated to inhibit the formation and progression of new psoriatic lesions following an injury to healthy skin.

## Abbreviations

ACKR2: atypical chemokine receptor 2
MAPK: mitogen-activated protein kinase
mS100a7a15: mice S100A7 and S100A15
NGF: nerve growth factor
NMDA: N-methyl-d-aspartate
NMDAR: NMDA receptor
PAR: proteinase-activated receptor
p75NTR: p75 neurotrophin receptor
RAGE: receptor of advanced glycation end product
STAT3: signal transducer and activator of transcription 3
TrkA: tyrosine kinase A
UEA I: Ulex europaeus agglutinin
VEGF: vascular endothelial growth factor
γδT17: IL-17 producing γδ T
